# Negative Regulation of Grb10 Interacting GYF Protein 2 on Insulin-Like Growth Factor-1 Receptor Signaling Pathway Caused Diabetic Mice Cognitive Impairment

**DOI:** 10.1371/journal.pone.0108559

**Published:** 2014-09-30

**Authors:** Jing Xie, Qianping Wei, Huacong Deng, Gang Li, Lingli Ma, Hui Zeng

**Affiliations:** 1 Department of Geriatrics, The First Affiliated Hospital of Chongqing Medical University, Chongqing, China; 2 Department of Endocrinology, The First Affiliated Hospital of Chongqing Medical University, Chongqing, China; 3 Department of Mental Health, The Mental Health Center of Jiulongpo District, Chongqing, China; Inserm U837, France

## Abstract

Heterozygous *Gigyf2* ^+/−^ mice exhibits histopathological evidence of neurodegeneration such as motor dysfunction. Several lines of evidence have demonstrated the important role of insulin-like growth factor-1 receptor (IGF1R) signaling pathway in the neuropathogenic process of cognitive impairment, while decreased Grb10-Interacting GYF Protein 2 (GIGYF2) expression can alter IGF1R trafficking and its downstream signaling pathways. Growth factor receptor-bound protein 10 (Grb10), a suppressor of IGF1R pathway, has been shown to play a critical role in regulating diabetes-associated cognitive impairment. It remains unknown whether endogenous GIGYF2 expression contributes to the development of diabetes-associated cognitive impairment. Using streptozotocin (STZ)-induced diabetic mice model, we first demonstrated that a significantly increased level of GIGYF2 expression was correlated with a significant decrease in the expression of phosphorylated IGF1R as well as the phosphorylation of AKT and ERK1/2, two signaling pathways downstream of IGF1R, in the hippocampus of diabetic mice. On the contrary, in situ knockdown of GIGYF2 expression in hippocampus resulted in increased expression of phosphorylated IGF1R expression and correspondingly reversed the down-regulation of ERK1/2 phsophorylation but had no obvious effect on Grb10 expression. Functionally, knockdown of GIGYF2 expression markedly ameliorated diabetes-associated cognitive dysfunction as well as the ultrastructural pathology and abnormal neurobehavioral changes. These results suggest that increased expression of GIGYF2 might contribute to the development of diabetes-associated cognitive disorder via negatively regulating IGF1R signaling pathway. Therefore, down-regulation of GIGYF2 expression may provide a potential novel approach to treat diabetes-associated cognitive impairment caused by aberrant IGF1R signaling pathway.

## Introduction

Numerous studies have shown that diabetic patients present a high risk of developing cognitive disorders [1], [2]. Nowadays, diabetic encephalopathy is recognized as one of the most important complications of diabetes, which encompasses functional impairment of cognition, cerebral signal conduction, neurotransmission and synaptic plasticity, and underlying structural brain abnormalities [1], [2].

Accumulating evidence indicates that insulin-like growth factor-1 (IGF1) acts as a homeostatic modulator for normal brain functionality and synaptic plasticity [3]–[5], and the loss of IGF1 activity caused by diabetes may contribute to cognitive impairment [6]. Most biological functions of IGF1, including its anti-apoptotic function, are mediated by the insulin-like growth factor-1 receptor (IGF1R) [7], [8]. Studies have shown that growth factor receptor-bound protein 10 (Grb10) can interact with tyrosine-phosphorylated growth factor receptors such as IGF1R and insulin receptor (IR) and serve as an endogenous negative regulator of IGF1R signaling [9], [10]. The interaction between BPS domain of Grb10 and IGF1R could directly inhibit IGF1R substrate phosphorylation [11], and decreased the levels of Grb10 expression below normal levels resulted in augmented IGF1 activation of Akt and ERK1/2 [9]. However, the N-terminally truncated Grb10 (BPS-SH2) shows no effect on receptor phosphorylation or glucose uptake, implying that the N-terminal domains of Grb10 is essential to its regulatory effect on IR signaling [12]. Recent studies via yeast two-hybrid screening have demonstrated that the N-terminus of Grb10 interacts with GYF proteins (GIGYF1 and GIGYF2), which are two novel and homologous proline motif binding proteins. The GIGYF1 protein can be recruited to the activated insulin and IGF1 receptors through binding to the N-terminus of Grb10 [13]. Subsequent studies using GIGYF2 null mice models showed that GIGYF2 gene disruption in mice led to inhibition of IGF1-stimulated IGF1R tyrosine phosphorylation and consequently, the manifestation of neurodegeneration [14]. Those findings suggest that Grb10 and GIGYF2 may act cooperatively to regulate IGF1R signaling. In addition, a high level of GIGYF2 expression is presented in the pancreas and testis as well as brain (including the hippocampus) of adult mouse, thus supporting a vital role of GIGYF2 in the regulation of IGF1R signaling in the central nervous system (CNS) [15]. Most recently, several lines of evidence have shown that GIGYF2 gene mutations are closely linked to human familial Parkinson's disease [16]–[18], one of the most common neurodegenerative disorders, thus further supporting the notion that GIGYF2 may play a critical role in neuronal degradation in CNS.

We have recently reported that a continuous hyperglycemia condition led to an increased expression of endogenous GRB10 in the hippocampus of rats with diabetic encephalopathy, which might cause damages to nerve function such as cognitive impairment [19]. In addition, Saenger *et al.* have reported that the insulin/IGF1 signaling pathways were implicated in dysregulated synaptic maturation and might play a key role in brain ageing and dementia as well as in learning and cognitive functions in rodent models [20]. However, the pathophysiological function of GIGYF2, particularly its role in the aberrant IGF1R signaling pathway in diabetes, remains largely unknown. In the current study, we first examined the level of GIGYF2 expression in hippocampus of diabetic mice and then used lentiviral vector-mediated delivery of short hairpin RNA (shRNA) to knockdown GIGYF2 expression to observe changes in animal behavior and ultrastructural pathology. The results suggest that altered GIGYF2 expression in the hippocampus of diabetic mice might affect IGF1R signaling pathway and subsequently improve cognitive performance.

## Materials and Methods

### Ethics Statement

All animals used in the study were handled according to the International Guiding Principles for Biomedical Research Involving Animals of the Council for International Organizations of Medical Sciences. Animal experiments were approved by the Committee on the Ethics of Animal Experiments of Chongqing Medical University. In brief, animals were fed with a nutritious standardized diet and with unrestricted access to the distilled water under clean circumstances at the Laboratory Animal Centre of Chongqing Medical University (Chongqing, China), and maintained on a constant 12 h: 12 h light/dark cycle. All mice were deeply anesthetized with an intraperitoneal injection of 3% chloral hydrate before sacrifice by decapitation.

### Animal models

Male C57BL/6 mouse (6–7 weeks old, weighing 20–22 grams) were purchased from the Third Military Medical University Animal Center (Chongqing, China). After a week of acclimation, all animals were starved for 8 hours, and then three-fifths of the mice were randomly selected for a single intraperitoneal injection of streptozotocin (STZ, 180 mg/kg; Sigma-Aldrich, USA) to induce diabetes as experiment group. STZ was dissolved in 0.1 M sodium citrate-hydrochloric acid buffer solution (pH 4.5). The remaining mice were injected with an equal volume of buffer solution without STZ as control group. Three days later, glucose in fasting blood collected from the tail vein was measured using a strip-operating blood glucose sensor (Accu-Check Aviva, Roche Diagnostics, Basel, Switzerland). Mice with a blood glucose level of 16.7 mmol/L or above were diagnosed as diabetes [21]. Afterwards, the blood glucose and body weight were measured once a week. Those mice in the experiment group were further randomly divided into three groups: diabetes mellitus (DM), sham-knocked down (DM+0), and the test (DM + shRNA) groups. Those mice in the control group were randomly divided into two groups: control (con) and con + shRNA group. Each group had 12 mice.

### GIGYF2-shRNAconstructs and Lentiviral vector production

GIGYF2-shRNA is a Mouse pGreenPuro lentiviral shRNA clone [22] obtained from System Biosciences (California, USA). The shRNA was packaged into pseudoviral particles and stored at −80°C to keep stability and full biological activity. The classic lentiviral vectors (RSV.cPPT.hCMV.cGFP.Wpre) carried a built-in green fluorescent protein (GFP), which was used as a tracer in the neurons. It was packaged using calcium phosphate transfection of 293 T cells [23]. Viral particles were collected and concentrated with a titer no less than 1×10^10^ transducing units (TU)/ml. For the *in vivo* experiments, 8% glycerol is required for long-term storage, which can be omitted from the media during plasmid preparation [24].

### Stereotaxic surgery

One week after STZ injection, the mice were anaesthetized with an intraperitoneal injection of 1% pentobarbital sodium (Sigma) (5 mg/100 g). To knockdown GIGYF2 expression in the hippocampus, the lentivirus expressing GIGYF2-shRNA was implanted into Cornu Ammonis area 1 (CA1) region on each side of the hippocampus. The stereotaxic coordinates were determined from a mouse brain atlas [25] as −2.3 mm posterior to bregma, −2.0 mm or 2.0 mm lateral to the midline and 1.8 to 2.0 mm ventral of the dorsal surface of the skull. The sham-knockdown group of mice was also injected with the same dose of lentivirus without GIGYF2-shRNA. All mice received an intrahippocampal injection of 1.0 µl virus per side delivered over 4 minute (0.25 µl/min). The syringe was left in place for 1 min after each injection and then was slowly withdrawn [26].

### Morris Water Maze (MWM)

The MWM was adapted from Barron *et al.* [27] and Gupta *et al.* [28]. Each step of the test was performed in a circular pool (diameter 120 cm) with a circular platform (diameter 10 cm). The maze was surrounded by a black curtain. There were four markers on the edge for location, and the pool was divided into four quadrants according to the entrance markers. Milk powder was used to make the water opaque, and the water temperature was kept between 23±1°C [29]. The platform was placed in one quadrant of the pool (1 cm below the water surface) and unaltered throughout the pre-training trials.

In the spatial acquisition trials, the mice were put to face the wall and then into the water at four starting positions and given 90 seconds (sec) to find the hidden platform. Each mouse was trained with four trials per day. Latency to find the platform (escape latency) was recorded on each trial. Mice were allowed to remain on the platform for 10 sec after reaching. If mice failed to find the platform within 90 sec, the trial was terminated and mice were guided to the platform and remained on it for 10 sec, and then put back into cages.

In the probe trial, the platform was removed. This trial was designed with a cut-off time of 60 sec. The frequency of mice swimming across the site where the platform was placed (platform crossings), and the time spent in the target quadrant was recorded [30]. After finishing one classical MWM test, the location of the platform was changed.

### HemateinEosin and Immunohistochemistry stain

Ten weeks after STZ injection, the mice were deeply anaesthetized with an intraperitoneal injection of 3% chloral hydrate and then transcardially perfused with 4% paraformaldehyde in phosphate buffer saline (PBS). The brains were removed and immersed into 4% paraformaldehyde for 24 hour at 4°C and then embedded in the paraffin. Paraffin-embedded sections of hippocampus were cut on vibratome at a nominal thickness of 5 µm. Tissue sections were subjected to dewaxing, dewatering and washed in PBS, and then treated with 10 mmol/L sodium citrate buffer (pH 6.0–6.3), heated in a microwave oven for 20 min at 92–98°C for antigen retrieval and incubated in 0.3% hydrogen peroxide for 15 min. After washing in PBS, tissue sections were blocked in 5% normal goat serum and 0.3%Triton X-100 in PBS for 30 min at 37°C, followed by incubation with the primary antibody solution (GIGYF2 antibody, 1∶150 dilution) (Santa Cruz Biotechnology Inc., CA, USA) overnight at 4°C. After washing extensively in PBS, tissue sections were incubated with a solution of 0.1% BSA containing biotinylated goat anti-rabbit secondary antibody (dilution 1∶200) at 37°C for 60 min, followed by incubation with in avidin-biotin horseradish peroxidase complex (Vector Laboratories, Burlingame, CA, USA) at 37°C for 30 min. After extensive washing with PBS, tissue sections were incubated in a 3, 30-diaminobenzidine solution (Sigma) until the development of a brown color [31]. At last, tissue sections were re-stained with haematoxylin, air dried and mounted with mounting medium. The pictures were collected on Olympus PM 20 (Olympus, Tokyo, Japan), and the density was measured by Image-Pro Plus, version 6.0 (Media Cybernetics, Inc., Silver Spring, MD, USA).

### Transmission electron microscopy (TEM)

Brain tissues were perfused with 2% glutaraldehyde perfusate (25% glutaraldehyde and 0.2 M phosphate buffer with 3 mM MgCl_2_, pH 7.4), followed by fixation with 4% glutaraldehyde perfusate. To observe the possible changes in synaptic and other ultrastructures, the sections for electron microscopy contained either the upper or the middle third of the CA1 stratum radiatum of the hippocampus [32]. The quantity of the spine density was determined by stereological techniques using the Physical Disector (Disector Countor, version 1.0; Department of Mechanics and Engineering Science, Peking University, Peking, China) [33].

### Real-time qRT-PCR

Ten weeks after STZ injection, the mice were deeply anaesthetized with an intraperitoneal injection of 3% chloral hydrate and then directly decollated on the ice to obtain hippocampus, which was rapidly separated and stored in liquid nitrogen. Total RNA from the hippocampus tissues was extracted using RNeasy Mini kit (Qiagen, Mississauga, ON, Canada) according to manufacturer's instructions. The RNA concentration and purity was measured using a NanoDrop 2000 c (Thermo Fisher Scientific Inc., Waltham, MA, USA). Pure RNA had an A260/A280 ratio of 1.8 and 2.0. cDNA was synthesized from mRNA using the PrimeScript RT Reagent kit (Takara Bio Inc., Otsu, Japan). Real time RT-PCR was performed using primer set for mouse target gene. The primers for real time RT-PCR were designed and synthesized by Sangon Biotech (Shanghai, China). Gene sequences of primers were as follows: GIGYF2 (forward primer, 5′-CTGTCGCCTCCTGTTCCTACT-3′; reverse primer: 5′- CTCTTCATCATCTGGCTCTGTG-3′); Grb10 (forward primer, 5′- GTGAAAGAGGTAGGACGCAAGT-3′; reverse primer: 5′-TCCAGCAATCAGGTAGAAGATG-3′); IGF1R (forward primer, 5′-GACTCGGATGGCTTCGTTATC-3′; reverse primer: 5′- CGATGGTTTTCGTTTTCTTCTC-3′). Each real-time PCR reaction was amplified with SYBR Premix Ex TaqTM II (Takara Bio Inc., Otsu, Japan) using a Bio-Rad CFX 96 Real Time System (Bio-Rad, Hercules, CA). The reaction mixtures contained: 200 ng of template, 0.8 µl of forward primer, 0.8 µl of reverse primer, and 10 µl of SYBR Premix Ex Taq (Tli RNaseH Plus). These mixtures were heated at 95°C for 3 min, 40 cycles of 95°C for 5 sec, 58°C for 30 sec, and 72°C for 30 sec. The comparative threshold cycle (Ct) for quantitative gene expression between target gene and β-actin was analyzed by Bio-Rad CFX Manager software (Bio-Rad, Hercules, CA). The relative change of gene expression was calculated with the 2^−ΔΔCt^ equation.

### Western blot analysis

The hippocampus tissues from mice were homogenized using a protein extraction kit (Beyotime Institute of Biotechnology, China) in 50 mM Tris (pH 7.4), 1% Triton X- 100, 1% sodium deoxycholate, 150 mM NaCl, 0.1% SDS, 1 mM PMSF and protease inhibitors. The tissue lysates were centrifuged at 12,000 rpm for 20 min at 4°C and the supernatant were collected to determine the protein concentrations by a bicinchoninic acid protein assay (Beyotime Institute of Biotechnology, China). Western blotting was performed as described previously [34]. Membranes were reprobed with an antibody specific against β-actin as an internal control. The semi-quantitative analysis of the bands was performed using Quantity One software version 4.6.2 (Bio-Rad, Hercules, CA, USA). The specific primary antibodies included: a rabbit polyclonal antibody for GIGYF2 (1∶150; Santa Cruz Biotechnology Inc., CA, USA), Grb10 (1∶200; Santa Cruz Biotechnology Inc.), IGF1R (1∶1000; ImmunoWay Biotechnology Inc., Newark, DE, USA), phospho-IGF1R (Y1161) (1∶1000; ImmunoWay Biotechnology Inc.), Akt (1∶1000; ImmunoWay Biotechnology Inc., Newark, DE, USA, YT0176), Phospho-Akt (S473) (1∶1000; ImmunoWay Biotechnology Inc., Newark, DE, USA, YP0864), ERK1/2 (1∶1000; ImmunoWay Biotechnology Inc., Newark, DE,USA,YT1623), and Phospho-ERK1/2(T202/Y204) (1∶1000; ImmunoWay Biotechnology Inc., Newark, DE, USA, YP1197), and a mouse monoclonal antibody for β-actin (1∶3500; Anbo Biotechnology Inc., San Francisco, USA).

### Statistical analysis

All results were analyzed using SPSS 19.0 (SPSS Inc., Chicago, IL, USA) and presented as the mean ± SEM. One-way analysis of variance (one-way ANOVA) was conducted. If a significant difference was found, a Bonferroni or Tamhane's T2 post-hoc analysis was conducted to determine which groups differed significantly according to the equal variance criterion. Repeated measure analysis of variance was used in Morris water maze test. All statistical tests were two-sided with significance set at *p*<0.05.

## Results

Since operative wounds can also influence animal behaviors, we did then performed the classic MWM test to assess the parameters associated with animal behavior changes such as exploratory activity, spontaneous locomotion, anxiety and reference memory performance. The results indicated that surgery did not have any obvious effects on those indices, thus suggesting that such changes in these indices might be due to the chronic hyperglycaemic conditions.

### Effect of hyperglycemia and GIGYF2-shRNA on body weight

Different groups of mice had similar body weight and blood glucose levels before STZ injection. One week after STZ injection, the level of blood glucose was significantly increased in diabetic groups (DM, DM +0 and DM + shRNA) (*p*<0.01, Fig. 1B), suggesting the successful induction of diabetes in those mice. During the whole experiment, the hyperglycemia condition in diabetes was persisted (Fig. 1B), and typical symptoms of diabetes (disproportionate thirst, intense hunger, frequent urination and unusual weight loss) were occurred. Diabetic mice were fatigue, irritability or indifference. One week after STZ injection, the weight of diabetic mice was significantly lower than that of non-diabetic groups (con and con + shRNA) (*p*<0.01, Fig. 1A). All diabetic groups showed a slow weight gain during the whole experiment, and had a significant lower body weight than that of non-diabetic groups in ten weeks after STZ injection (*p*<0.01, Fig. 1A). Even though DM + shRNA group gained more weight than that of DM and DM +0 groups during the whole experiment, the difference was non-statistically significant (*p* = 0.142).

**Figure 1:** Body weight (A) and blood glucose levels (B). The body weight (A) and blood glucose levels (B) of C57BL/6 mice were measured once a week. Blood samples were collected from the tails of mice under fasting condition. The body weight was measured in gram, and the blood glucose was measured using a strip-operating blood glucose sensor. The data expressed as the mean ± SEM (n = 12). Abbreviations: con: normal control group; DM: diabetes mellitus group; DM +0: diabetes mellitus sham-knocked down group; con + shRNA/DM + shRNA: control/diabetes mellitus GIGYF2-knockdown group.

### Viral-mediated GIGYF2 knockdown and its effect on IGF1R signaling

The levels of GIGYF2 expression and its related genes (Grb10, IGF1R) in hippocampus tissue were detected by real time- PCR and Western blotting, respectively. We found that DM and DM +0 group, but not DM + shRNA group, had a significant increase in the level of GIGYF2 expression compared to control group (*p*<0.05, Fig. 2A and 3A). These results demonstrated that GIGYF2 expression was specifically knocked down at both mRNA and protein levels by site-application of special GIGYF2-shRNA. As for Grb10 expression, there were no obvious differences among the three diabetic groups (*p* = 0.172, Fig. 2B and 3B), but it was higher than that of two non-diabetic groups (*p*<0.05). Similarly, the levels of IGF1R expression in the three diabetic groups were not obviously different (*p* = 0.651, Fig. 2C and 3C), but were significantly decreased compared to two non-diabetic group (*p*<0.05). Nevertheless, the expression level of IGF1R phosphorylation (phosph-IGF1R, the phosphorylation site of Tyr1161) was significantly increased in DM + shRNA group as compared with that in DM and DM +0 groups (*p*<0.05, Fig. 3D).

**Figure 2:** The expression levels of target gene mRNA. The levels of Grb10 Interacting GYF Protein 2 (GIGYF2) mRNA (A), growth factor receptor-bound protein 10 (Grb10) mRNA (B) and insulin-like growth factor-1 receptor (IGF1R) mRNA (C) were detected by using the real-time polymerase chain reaction and quantified from three independent experiments, and average levels in septum of each group mice were shown in the graphs. Regulation of Grb10 Interacting GYF Protein 2 (GIGYF2) levels using a lentiviral vector carrying GIGYF2-short hairpin (sh) RNA. Histogram represents the gene expression of target genen, compared to the control group. The data expressed as the mean ± SEM (n = 3). (*p<0.05, **p<0.01 *vs* con; ^#^ *p*<0.05, *vs* DM + shRNA) Abbreviations: con: normal control group; DM: diabetes mellitus group; DM +0: diabetes mellitus sham-knocked down group; con + shRNA/DM + shRNA: control/diabetes mellitus GIGYF2-knockdown group.

**Figure 3:** The expression levels of target protein. The protein levels of Grb10 Interacting GYF Protein 2 (GIGYF2) (A), growth factor receptor-bound protein 10 (Grb10) (B), insulin-like growth factor-1 receptor (IGF1R) (C) and phosphorylated IGF1R (D) were measured by using western blotting and quantified from three independent experiments, and average levels in septum of each group mice were showed in the graphs. Band intensities of phosphorylated IGF1R were normalized to total IGF1R. Except of phosphorylated IGF1R, band intensities were normalized to β-actin. The data expressed as the mean ± SEM (n = 3). (*p<0.05, **p<0.01) Abbreviations: con, normal control group; DM, diabetes mellitus group; DM +0: diabetes mellitus sham-knocked down group; con + shRNA/DM + shRNA: control/diabetes mellitus GIGYF2-knockdown group.

To further elucidate the mechanism of GIGYF2 involved in the regulation of IGF1R-mediated signaling pathways, the levels of total and phosphorylated serine/threonine kinase (phosph-Akt, the phosphorylation site of Ser473), extracellular signal-regulated kinase (phosph-ERK1/2, the phosphorylation site of Thr202/Tyr204) were examined by Western blot analysis. As shown in Fig. 4A, the total levels of either Akt or ERK1/2 were similar between control and diabetic mice. Nevertheless, the phosph-AKT to AKT ratios was significantly decreased among the three diabetic groups as compared to control group (*p*<0.01), and no obvious differences existed between DM + shRNA group and DM group (*p* = 0.307), nor between DM +0 group and DM group (*p* = 0.999). The phospho-ERK1/2 to ERK1/2 ratio was also decreased in the DM group (*p*<0.01) and DM +0 group (*p*<0.01) (Fig. 4B) as compared to control, but disruption of GIGYF2 gene expression in hippocampus of diabetic mice resulted in a significant increase in the levels of phosphorylated ERK1/2 as compared to DM group (*p*<0.05), and the ratio was comparable to that of normal control mice (*p* = 0.823).

**Figure 4:** The expression levels of Akt and ERK1/2. The protein levels of serine/threonine kinase (Akt) (A), extracellular signal-regulated kinase (ERK1/2) (B) were measured by Western blotting. The graphs showed the relative density of phosphorylated AKT or ERK1/2 to the total AKT or ERK1/2. The bars represented results from three independent experiments. Band intensities of phosphorylated protein were normalized to total protein. The data expressed as the mean ± SEM (n = 3). (**p<0.01 *vs* con) Abbreviations: con, control group; DM, diabetes mellitus group; DM +0: diabetes mellitus sham-knocked down group; DM + shRNA: diabetes mellitus GIGYF2-knocked down group.

### Effect of decreased expression of GIGYF2 on cognitive function

Effect of STZ and stereotaxic surgery on the MWM was negligible (Fig. 5A_a, b_, B and C). No significant differences in the mean escape latency (Fig. 5A_a, b_), platform crossing (Fig. 5B) and time in target quadrant (Fig. 5C) among the groups were observed when the diabetes was induced just one week after STZ injection. The water maze experiment was executed once more at one week after surgery, and there were no significant differences among different groups, too. Ten weeks after surgry, the mean escape latency of DM and DM +0 groups was apparently increased and both had a significant difference compared to control group (both *p*<0.05, Fig. 5A_c_). The results indicate that the spatial memory was impaired in diabetic mice, which could be used as an indicator of diabetic encephalopathy. Meanwhile, the mean escape latency of DM + shRNA group was not increased and showed no obvious difference compared to control group (*p* = 0.376), but significant lower than that of DM and DM +0 groups (*p*<0.05). These findings suggest that GIGYF2-shRNA or specific knockdown of GIGYF2 could attenuate the spatial learning impairment associated with diabetes. Regarding probe trials, the time in target quadrant of DM and DM +0 group was declined and had a similarly significant difference compared to the control and DM + shRNA groups (*p*<0.01, Fig. 5C). However, no differences were observed between DM + shRNA group and control group (*p* = 0.978, Fig. 5C). In addition, platform crossing was not significantly different between DM group and DM + shRNA group (*p* = 0.062, Fig. 5B). This might be due to the limitation of platform crossings, e.g. variable and often a low frequency of occurrence. In addition, crossover undercounting might occur depending on tracking software [30].

**Figure 5:** The results of Morris water maze (MWM) test. Morris water maze (MWM) test was performed before intrahippocampal injection surgery, 1 week after surgery and 10 weeks after surgery in adult male mice. Learning acquisition curve showing the effects of streptozotocin and a single surgery on spatial learning (A_a, b_) and the protective effects of Grb10 Interacting GYF Protein 2 (GIGYF2)-short hairpin (sh) RNA (A_c_) using the mean escape time to reach the hidden platform (escape latency) over consecutive trials in the MWM task. For the probe trials, the platform crossings (B) and time spent in the target quadrant (C) was recorded. Data are expressed as the mean ± SEM (n = 12 per group). (*p<0.01 *vs* con; ^#^ *p*<0.01 *vs* DM + shRNA) Abbreviations: con: normal control group; DM: diabetes mellitus group; DM +0: diabetes mellitus sham-knocked down group; con + shRNA/DM + shRNA: control/diabetes mellitus GIGYF2-knockdown group.

### HemateinEosin and Immunohistochemical staining in the hippocampus

Continuous exposure to hyperglycemia (DM and DM +0 group) led to changes in cell morphology, including a decrease in neuron numbers, an increase in neuron apoptosis and disordered cell arrangement in the pyramidal cell layer of hippocampus. The morphology of cell was not significantly altered in the hippocampus of GIGYF2-knockdown diabetic mice (Fig. 6A). Immunohistochemical staining showed that GIGYF2 was located in cytoplasm or on membrane as reported in a recent study [15]. Quantitative analysis showed that the level of GIGYF2 protein expression in DM + shRNA group was significant lower than that of DM and DM +0 groups (*p*<0.05, Fig. 6B and C), but had no significant difference compared to the control group (*p* = 0.289). The level of GIGYF2 expression of DM and DM +0 group was comparable (*p* = 0.161).

**Figure 6:** Haematoxylin and eosin staining (HE) of hippocampal tissue. Arrows show senescent neurons (A, inset windows) and cell disorder arrangement (A) in the DM group compared to the healthier hippocampal neurones in the DM + shRNA group and the normal ones in the con group. Immunohistochemistry of hippocampus tissue indicated the place and expression levels of Grb10 Interacting GYF Protein 2 (GIGYF2). Integrated optical density (IOD) values were measured by Image-Pro Plus, version 6.0, and expressed as the mean ± SEM (n = 3) of two independent experiments. (*p<0.05 *vs* con; ^#^ *p*<0.05 *vs* DM + shRNA) Abbreviations: con: normal control group; DM: diabetes mellitus group; DM +0: diabetes mellitus sham-knocked down group; DM + shRNA: diabetes mellitus GIGYF2-knockdown group.

### Changes of tissue ultrastructure in the hippocampus

As expected, the results of electron microscopy indicated that the number of spine synapses in the CA1 region of hippocampus of DM + shRNA group was significant greater than that of the DM group (*p*<0.05, Fig. 7) because of a significant loss in the number of spine synapses in DM group. And there was no obvious difference between DM + shRNA group and control group (*p* = 0.177).

**Figure 7:** Morphology and spine synapse density. Morphologically intact synapse (arrows) are indicated and do not change by the effect of Grb10 Interacting GYF Protein 2 (GIGYF2)-short hairpin (sh) RNA. By contrast, in the DM group, hyperglycaemia results in a significant decrease in synapse density and swollen axons at 10 weeks after streptozotocin injection. Values of the quantity of the spine density are determined by pictures of 8000 times amplification using stereological technique in the Disector Countor, version 1.0 software, and the data are expressed as the mean ± SEM (n = 3). (*p<0.05 *vs* con; ^#^ *p*<0.05 *vs* DM + shRNA) Abbreviations: con: normal control group; DM: diabetes mellitus group; DM +0: diabetes mellitus sham-knocked down group; DM + shRNA, diabetes mellitus GIGYF2-knockdown group.

## Discussion

In the present study, we investigated the effects of GIGYF2 on cognitive function using streptozotocin (STZ)-induced diabetic mice. Our results revealed that the level of GIGYF2 expression was significantly up-regulated in hippocampus tissue of diabetic mice (Fig. 2A and 3A), which is correlated with manifestations of diabetes-associated cognitive impairment (Fig. 5). Moreover, diabetic mice with hippocampus-specific knockdown of GIGYF2 expression (DM + shRNA group) showed less cognitive impairment and less pathological ultrastructure changes than other diabetic mice (DM and DM +0 groups), thus supporting the notion that GIGYF2 plays an important role in the development of diabetic encephalopathy. Meanwhile, we found that the level of total IGF1R expression (Fig. 2C and 3C) was significantly decreased, but the level of phosphorylated IGF1R and the level of phosphorylated ERK1/2 was significantly increased in DM + shRNA group. These findings suggest that GIGYF2 may contribute to cognitive disorder development possibly by negatively modulating the level of phosphorylated IGF1R and its downstream signaling pathways, and hippocampus-specific down-regulation of GIGYF2 is beneficial for neuroprotection in diabetic encephalopathy.

### Over-expression of GIGYF2 reduces cognitive function

A previous study has reported that GIGYF2 might also play a role in the regulation of trafficking of IGF1R in specific neuronal populations of the mammalian brains, including hippocampal pyramidal neurons [15]. The hippocampus is a brain area known to be important for learning and memory, especially vulnerable in Alzheimer's disease [35]. As a result of the unique localization of GIGYF2 expression in brain, we transduced GIGYF2-shRNA lentiviral vectors into the hippocampus by stereotaxic injections, aiming to achieve organ-specific knockdown of the target gene in the brain of mice. The efficiency of hippocampus-specific knockdown of GIGYF2 expression was verified by real time-PCR and western blotting analysis, showing that the stereotaxic injection of GIGYF2-shRNA lentiviral vectors significantly abrogated the expression of endogenous GIGYF2 in diabetic mice.

In the water maze test, all groups exhibited a normal spatial memory when the surgery had just been executed. However, when the test was performed again nine weeks later, the diabetic mice without shRNA injection (DM and DM +0 groups) performed more poorly than DM + shRNA and control groups (Fig. 5A_c_ and B), which was in accordance with the level of GIGYF2 expression in each group (Fig. 2A and 3A) and the changes in behavior and cognitive impairment in the experimental diabetes [36]. These findings suggest that the decline of temporal memory and learning abilities during continued exposure to high glucose [37] is significantly alleviated after the down-regulation of GIGYF2 in brain. Moreover, our results showed that down-regulation of GIGYF2 could reduce changes of cell morphology such as neuronal apoptosis and disordered arrangement (Fig. 6A). Additionally, the improvement in pathological ultrastructure changes in the hippocampus suggests that the low expression level of GIGYF2 in diabetic mice is beneficial to the homeostatic regulation of synaptic functions.

### Over-expression GIGYF2 inhibited IGF1R signaling pathway in the brain

IGF1R is known to be a membrane-associated multifunctional tyrosine kinase (TK) receptor implicated in several basic biological events, such as cell proliferation, differentiation and protection from apoptosis [38]–[40]. In the brain, IGF1R is activated by two ligands (IGF1 and IGF2), and IGF1 has been shown to play a role in synaptic plasticity and acts as a potential treatment target for the cognitive dysfunction [5]. The dysregulation of synaptic maturation and disruption of IGF1 downstream signaling pathways are both involved in some of these cognitive disorders, including diabetic encephalopathy [20], [41].

Giovannone *et al* have reported that the level of phosphorylated IGF1R was decreased in the mice that had decreased expression level of GIGYF2 gene [14]. However, our present studies showed that the level of total IGF1R (Fig. 2C and 3C) and phosphorylated IGF1R (Fig. 3D) was significantly decreased in hippocampus of diabetic mice that had significantly increased expression level of GIGYF2 (Fig. 3A). In another group of diabetic mice that received shRNA injection (DM + shRNA group), the phosphorylated IGF1R level (Fig. 3D) and GIGYF2 expression (Fig. 3C) were both comparable to normal level in hippocampus, but the level of total IGF1R in hippocampus of these mice was still significantly decreased (Fig. 2C and 3C). These results indicate that both the increased and decreased expression level of GIGYF2 may lead to altered levels of phosphorylated IGF1R, then possibly inhibit IGF1R signaling pathway.

It is well established that IGF1 receptor phosphorylation mediated by IGF1 stimulation leads to the activation of two distinct downstream signaling pathways, which are the src homology 2/mitogen-activated protein kinase (Shc/MAPK) pathway and the phosphatidylinositide 3-kinase/serine/threonine kinase (PI3K/Akt) pathway. Previous studies have demonstrated that the expression level of IGF1 and IGF1R decreased in brain tissue of diabetes [42], [43], and disruption of the GIGYF2 gene in mice led to a decrease in IGF1-stimulated IGF1R tyrosine phosphorylation but an augmentation in ERK1/2 phosphorylation [14]. However, the increased expression of GIGYF2 in HEK293T cells augmented IGF-1-induced ERK1/2 activation, but did not modulate IGF1R or Akt activation [15]. Herein, we further examined the effects of downregulation of GIGYF2 expression in diabetic mice on the activation of AKT and ERK1/2 (Fig. 4) and found that the decreased levels of phosphorylated Akt and ERK1/2 were correlated with the decreased level of phosphorylated IGF1R in diabetic mice, while down-regulation of GIGYF2 expression to normal endogenous levels in hippocampus of diabetic mice augmented ERK1/2 activation (Fig. 4B), but did not modulate Akt activation (Fig. 4A). These results suggest that GIGYF2 may have a role in the regulation of IGF1R and its downstream ERK1/2 signaling pathway, but not Akt signaling pathway.

### Relationship between GIGYF2 and cell apoptosis

Of note, recent studies have demonstrated that IGF1 resistance in the central nervous system reduces Amyloid-β accumulation and prevents premature death in a model of AD [44]. Postmortem investigations have revealed a decreased expression of cerebral IGF1R and insulin receptor substrate (IRS) proteins in patients with AD [45]. Similar changes in IGF1R signaling have been described in diabetes [46], suggesting that decreased IGF1/IGF1R signaling might be involved in the pathogenesis of both diabetes and AD. The conformational changes caused by the binding of IGF1 or IGF2 to IGF1R lead to autophosphorylation of the receptor. Then this autophosphorylationy of IGF1R leads to the phosphorylation of its downstream signaling intermediates such as insulin receptor substrate (IRS) and Shc [47], and activates the AKT and ERK1/2 signaling [48]. Activation of IGF1R signaling pathways protects cells from apoptosis via activiting IGF1R downstream signaling, with an associated increase in IGF1-mediated DNA synthesis [49], [50]. Our results showed that down-regulating the increased GIGYF2 expression to the normal level restored the decreased phosphorylation of IGF1R and the decreased phosphorylation of ERK1/2 to the normal level. This finding indicates that over-expression of GIGYF2 might lead to downregulation of IGF1R phosphorylation, and such effects could be abolished when the expression level of GIGYF2 was reduced to a normal level. Our current results showed that the over-expression GIGYF2 is correlated with an increase neuron apoptosis (Fig. 6 and 7). On the other hand, Giovannone *et al* have reported that the decreased expression level of GIGYF2 in mice resulted in neurodegeneration [14]. Together, these findings suggest that GIGYF2 may play a role in the regulation of cell apoptosis. However, further studies are warranted to explore the detailed mechanisms.

### Relatively independent effect of GIGYF2 and Grb10 on IGF1R signaling

It has been demonstrated that endogenous Grb10 might prevent phosphatase from accessing to the activated IGF1R [9]. GIGYF2, as an endogenous regulator of IGF1R signaling, was initially identified through its interaction with the N-terminus of Grb10 [11]. Interacting and co-localizing between GIGYF2 and Grb10 could promote ligand-induced ubiquitination of IGF1R, and then resulted in IGF1R degradation [15], [51]. Our previous studies have proved that the over-expression of Grb10 was harmful to cognitive function in diabetic rats, and a regulatory axis composed of IGF1/IR and the downstream Grb10 regulator had a role in regulating biological functions of the hippocampus [20]. In present study, we found that the level of Grb10 expression was significantly increased in the hippocampus of diabetic mice, which was consistent with our previous report [20]. However, disruption of GIGYF2 expression in hippocampus had no obvious effects on Grb10 abundance (Fig. 2B and 3B), indicating that GIGYF2 expression might have no obvious relationship with Grb10 expression. Previous observations showed that GIGYF2 may function at endosomes where the traffic and recycling are regulated by Rab4, a protein belonging to Rab protein family of small guanosine-5′-triphosphate (GTP)-binding proteins [15]. The Ridaifen B (RID-B), a tamoxifen derivative that potently inhibits breast tumor growth, can directly bind to GIGYF2 and subsequently inhibit GIGYF2-induced Akt phosphorylation [52]. Based on these findings, we can speculate that, in diabetic encephalopathy, the effect of GIGYF2 on IGF1R signaling is not only mediated by cooperation with Grb10, but also by interaction with some other molecules. Therefore, future studies are needed to further explore the molecular mechanisms underlying GIGYF2-mediated regulation of IGF1R and its downstream signaling pathway.

It is noteworthy that STZ-induced DM model in mice is not an optimal model, especially as the influence of STZ cannot be fully excluded. In the present study, the water maze experiment was executed when the acute diabetes was induced just one week after STZ injection in order to exclude the effect of STZ on cognitive function, and no significant differences in the mean escape latency, platform crossings and time in target quadrant were noticed among different groups (Fig. 5). These results have shown that all mice presented a normal spatial memory soon after STZ injection. Meanwhile, previous studies have successfully used this experimental diabetes model to investigate cognitive impairment and changes in behavior of diabetic animals [36], [53], [54].

## Conclusion

In conclusion, we have demonstrated that the level of GIGYF2 expression was significantly increased in the hippocampus under a continuous hyperglycemic condition and could be efficiently down-regulated by directly applying lentiviral vector-delivered GIGYF2 shRNA to the hippocampus *in vivo* using stereotactic technology. Our findings suggest that GIGYF2 may play an important role in the development of diabetes-associated cognitive impairment through modulating the phosphorylation of IGF1R and its downstream ERK1/2 signaling pathway, but not Akt signaling pathway. Down-regulation of GIGYF2 expression may provide a potential novel approach to treat diabetes-associated cognitive impairment caused by aberrant IGF1R signaling pathway.
